The article "Association between community psychological label and user portrait model based on multimodal neural network" was published in 2022. Journal: Front Psychol.

# Association between community psychological label and user portrait model based on multimodal neural network

**DOI:** 10.3389/fpsyg.2022.918274

**Published:** 2022-08-24

**Authors:** Hao Jiang, Xuehong Yin

**Affiliations:** ^1^School of Economics, Zhejiang Gongshang University, Hangzhou, China; ^2^School of Accounting, Zhejiang Gongshang University, Hangzhou, China

**Keywords:** user portrait, knowledge representation, multimodal neural network, community psychological label, correlation

## Abstract

By analyzing traditional deep learning multimode retrieval methods, an optimized multimode retrieval model based on convolutional neural network is established. This article proposes an innovative semi-supervised social network user portrait analysis model (UPAM) based on user portrait model, which integrates users’ social information and some known user attribute information (such as educational background and residence) into a unified topic model framework. Finally, a semi-supervised user portrait analysis method based on user social information and partial known user attribute information is proposed. According to the correlation of user attributes, the cross-validation method is used to train model prediction task and improve the prediction effect. In the first-level model, using a different model to extract the features in the user query, the basis of the second hierarchy model, Stacking is used to further integrate characteristics, finally realizing the attribute population forecast, and experimental verification showing the proposed model’s effectiveness in various attributes of a population.

## Introduction

With the advent of the information age, it is obvious that single-mode retrieval could not meet people’s demand for retrieval. Early multimodal retrieval mainly depends on the characteristics of manual annotation (Linden et al., 2021) and is essentially a single-modal retrieval, for example, in the Baidu image input text retrieval-related pictures, its return is the result of the image, but these results are in accordance with annotating text information, and at the same time the picture of the text annotations cannot be successfully retrieved. In this era of rapid information development, it is obviously impossible to label all the information one by one, which leads to the related research of multimodal retrieval. In addition to retrieval problems, another challenge of the data explosion era is how to store and manage these massive amounts of multimodal data effectively. Only the related work of storage and management can meet the requirements of retrieval speed and accuracy.

Data of different modes have their own underlying features. For pictures, the underlying features include color and texture, while for text, the underlying features include subject, predicate, object, and words, as well as tone of audio data. After years of research by relevant scholars, it can be concluded that there is a “semantic gap” between the high-level semantics and the low-level features of data, and at the same time, data of different modes are heterogeneous. Therefore, the key of multimodal data retrieval technology research is to bridge the “semantic gap” (Zheng et al., 2016), which is generally speaking finding out the internal correlation information between different modal data.

If the training is carried out only by users with attribute information, due to the limitation of data, the final model trained often does not have good generalization. If you abandon a large number of users whose attribute information is incomplete, it is undoubtedly a huge waste of data resources. Therefore, how to make use of the complete social network structure information and part of the known user attribute information to obtain a user portrait analysis model with stronger generalization ability has become a question to be answered. Semi-supervised learning is one of the most important learning techniques using unlabeled data. The core problem is to establish a reasonable relationship between the distribution of unlabeled data and learning objectives so as to use unlabeled data to assist in improving learning performance. Therefore, the expected goal of this article is to use semi-supervised method to model the user portrait analysis problem and obtain a user portrait analysis algorithm with high precision and strong generalization ability so as to achieve accurate prediction of user attribute values. The prediction performance of the proposed multimodal neural network algorithm is compared with that of the corresponding basic model. It is verified that the performance of the multimode neural network method is better than that of the basic model and the multimode neural network method has better generalization ability and prediction ability. Then, the user queries the names of people, place names, rare words, and other words in the word, as well as the polysemy phenomenon. The first part is the introduction, the second part is related work, the third part is the research on community psychological labeling model based on multimode convolutional neural network, the fourth part is example verification, and the fifth part is conclusion.

## Related work

Early multimodal methods relied on human labor to perform feature extraction operations. A joint graph normalized multimodal subspace learning algorithm is proposed. By integrating the inter-modal similarity and intra-modal similarity into the graph regularization term (Khalaf et al., 2020), the relationship between multimodal data and the relationship between the data within each mode can be better represented. Abstract relation between image and text data is established by analyzing the abstract relation between image and text data. Text features are represented by the topic model (Akbar et al., 2017; Murayama and Ohya, 2021), and image features are represented by the word vector of Scale Invariant Feature Transform features. A semantic generation model is proposed, which assumes that each modal data is conditionally independent of a particular concept, so the same semantic concept can be generated. Next, Gaussian distribution and random forest are used to predict the probability distribution of semantic correlation, which improves the accuracy of retrieval and ensures the computational efficiency (Li et al., 2020). This article analyzes and solves the problem of multimodal semantic association from the perspective of low-level multimodal data connection and high-level semantic space abstraction, and proposes a semantic connection model combining these two ideas. A learning algorithm related to supervised multimodal is proposed, which overcomes the shortcoming of relying on paired image text data (Su et al., 2021) and can learn multimodal representation of independent single-modal data. Generalized Search Trees feature is used for image data and word frequency feature is used for text data. A multimode adaptive autoencoder model is proposed, which consists of two single-mode adaptive autoencoders (Ho et al., 2018). By minimizing the reconstruction errors of the two autoencoders and the correlation errors of the multimodal data, the common correlation between the two aspects of the shape representation layer is modeled. In addition, a variety of modal data mappings from the original semantic space to the lower-level common subspace are established, and the corresponding constrained Boltzmann machine is used to maintain the original semantic association (WeiWei, 2020). Deep convolutional neural network is used to learn image feature representation and multilayer perceptron is used to learn text feature representation, and the connection between the two subnets is established by objective function. In multiple multimodal retrieval databases, it has been found that the retrieval model based on depth feature representation significantly improves the performance compared with the traditional manual feature-based method (Liu et al., 2019). Similarly, a two-way image and text retrieval model based on convolution is proposed (Rathi and Roy, 2018). Two convolutional neural networks are designed for image and text functions, and the two modal data are compared with the public space on the network to achieve multimodal retrieval. Deep learning in the field of multimodal retrieval provides an end-to-end learning solution that integrates the feature representation of the underlying public space into the framework and achieves multimodal feature extraction according to the features of the deep learning network structure. However, with the continuous growth of multimedia data, feature representation using deep learning is faced with problems such as large storage space and dimension, which affect the retrieval efficiency, so it could not adapt to large-scale multimodal data retrieval tasks.

Different from the first approach, the second approach focuses on the social relationship itself. There are some common assumptions in the field of social network analysis, for example, users with similar attributes are more likely to become friends, and users with friend relationships tend to have similar attributes (Williams et al., 2018). It is the basic assumption, user portrait researchers attempt to understand the social relationship itself, to excavate the potential link between people, to explain the potential factor for the formation of good friend relationship (e.g., education background, similar to that of similar geographic location, similar interests and hobbies, the same school), and according to the contact of the potential user image analysis. User portrait is a mathematical model of real users. In the whole mathematical model, its core is to describe the business knowledge system, and the business knowledge system is ontology, as a modeling tool that can describe the conceptual model of information system at the semantic and knowledge levels is a clear formal specification of shared conceptual model. Due to the complexity of ontology, a very simple implementation of one tag (Carhart-Harris et al., 2016) is often adopted in engineering so as to use the collection of tags to represent user portraits. What kind of label is used is different for different businesses and data sets, so the user profile is more business based. Current research does not specifically study the establishment of user portraits, but for different business scenarios, user portraits are modeled as features of the recommendation system (Jaime et al., 2018). The constructed user portraits are defined according to the specific application scenarios and data sets. User-generated content in social networks is often used for analysis to build content-based characteristics. It mainly focuses on user portraits in academic circles. The user portraits are modeled by expanding ontology (Shelef et al., 2016), in which four basic concepts, 29 attributes, and four relationships are defined. Users can fully represent a user interest preference characteristic, often the user interest preferences in research and engineering as a portrait of a dimension, and the users use a lot of research work by using data mining methods to mining network user interest preference: using the tag behavior of users to get implicit social chains has proved it is used as a good index of user interest (Kayser et al., 2015). It mainly focuses on the tweets sent by Twitter users, and Twitter is also concerned with the user portrait, which has established a word bag model for each user: the user portrait of users is established. The article uses the user portrait based on hashtags, entities, and topics to improve the diversity and accuracy of user portrait through rich semantics.

As the research on the correlation between the community psychological standard of network multimodal neural network and the user portrait model continues to be found, the behavioral characteristics of Twitter users are paid attention to and the user’s behavioral characteristics are proposed for the first time to predict user personality (Ludwin and Capstick, 2015). The study collected 50 tweets: nearly 2,000 tweets from users, and the basic information of users obtained through Twitter API. The characteristics of Twitter users mainly selected in this article include number of fans, number of followers, degree of network, number of “@” symbols, number of replies, number of “#” tags, number of links, and average number of words per tweet. In addition, to confirm that people’s language patterns can still predict personality on Twitter, LIWC tool and Mixed Reality Capture psychological tool are used to obtain the linguistic features of users’ tweets. In addition, the General Inquirer data set was used for sentiment analysis of each tweet as another dimensional feature (Jimenez et al., 2015). After extracting these features, this article uses machine learning algorithm to learn the regression model of personality so as to predict the user’s personality through the behavior characteristics of network users. In addition to increasing the tag data set, the research is more about extracting more features. For example, the study on Facebook data set, the application of Psychometric personality test based on Facebook (Miquel et al., 2017). The article obtained 58,466 users’ psychological personality test scores, basic information of users, and Facebook Likes. The article can predict users’ characteristics, including sexual orientation, clan, religion, political opinions, personality characteristics, intelligence, happiness, age, and gender. Some sources (Steiner et al., 2017; Solowij et al., 2018) mainly focus on the content characteristics of Sina Weibo users. The data set of this article selected 1,766 Sina Weibo users to obtain their Big Five personality score data and their Sina Weibo content. This article extracted the user’s text features, including six aspects of 168 dimensions: microblog statistical features (including total number of microblog, microblog word count); syntactic features (including the number of Chinese characters in each sentence, the proportion of declarative sentences); morphological features (including total number of emotional words, total number of greetings); character characteristics (total number of periods, colons, 23 special symbols); features of Sogou Factory thesaurus (divided into 13 categories); and LIWC features (88 dimensions). Existing studies select large and comprehensive features, considering all aspects of static and dynamic information, and can obtain more features through extraction to improve the accuracy of the prediction model. The main focus of this article is to explore and study the relationship between the community psychological criteria of multimodal neural network and user portrait model.

## Research on community psychological labeling model based on multimode convolutional neural network

### Optimization structure of multimode convolutional neural network community mental label

To ensure that the retrieval results are more accurate and comprehensive, it is necessary to have a large number of multimodal data stored in the database, so the multimodal data management module is also an indispensable part of the prototype system. In this module, user mode data upload and query operations are present. To compare the retrieval accuracy of different models, the multimodal retrieval system in this article has embedded two multimodal hash retrieval methods in the system. Users can select different models for feature extraction of uploaded multimodal data and can also select different parameters and hash code length. When entering the retrieval interface, the corresponding retrieval results will be returned according to the selected model. The structure is shown in Figure 1.

**FIGURE 1:** Structure diagram of multimodal neural network community psychological label optimization.

The data set collected a total of 1,034 Sina Weibo users. These users were invited to take the Big Five personality test using the 44-item Big Five Questionnaire to obtain the user’s Big Five personality score. The Big Five score is a positive whole number. The statistical information of the Big Five personality scores of 1,068 tested users is shown in Table 1.

**TABLE 1:** Statistical information of five personality scores of users.

Value	A	B	C	E	N
Minimum value	18	12	9	17	9
Maximum	43	46	39	48	38
Average	32.876	28.34	23.76	35.56	25.15
Standard deviation	5.028	5.82	5.58	6.32	5.46

After the initial setting of model parameters, input the text after word segmentation into the model, use Gibbs sampling to conduct cyclic sampling of model parameters, and estimate the parameters after reaching the set cyclic threshold. For the Latent Dirichlet Allocation (LDA) model, there is the concept of “document,” which corresponds to the Sina Weibo data in this experiment. In the experiment, each microblog is input as a “document.” The generated result of the LDA model is the probability distribution matrix of document topic, from which the probability distribution of the corresponding topic of each document can be obtained. In this experiment, after obtaining the document topic distribution, the topic corresponding to the maximum probability of each document is selected as the topic of this document so as to obtain the corresponding topic label of each document. Still existing in the output of the LDA model subject term probability distribution matrix, you can get from the distribution of each topic on the global term vectors probability distribution. To be able to artificially observe specific implications of each topic, each theme selected typically corresponds to the maximum probability of the first *n* words as the subject of key, which makes it easier to observe the meaning of each theme.

Calculated for the experiment of 1,034 users in its each post corresponding to the theme of the label and corresponding keywords were each topic and quantitative subject characteristics; for each user, the corresponding number of 500 Weibo is calculated under each topic, and then after normalized processing, the total number of Weibo under each topic by proportion of the total number of all the user microblogging was 534. Thus, feature extraction based on LDA topic model is completed.

Based on weight matrix W, this article defines the first-order transition probability between different nodes. The first-order transition probability refers to the transfer after step probability from the constructed neighbor figure arrived; in the same way, based on the first-order transfer probability can also through the matrix multiplication be easier to find as well as second-order transition probability matrix and the high-order probability transfer matrix. Formalized, P is assumed to be a first-order probability transition matrix, where the element Pk represents the probability of reachability from node 2 to node K, which can be defined as follows:


(1) $$p_{k}=W_{k}\,/\,\left(W_{1}+W_{2}\,\ldots +W_{k}\right)$$

Although the weight matrix W is symmetric, the probability transition matrix P is not necessarily symmetric because the regular terms are different from point to point.

The first-order probability transition matrix is directly represented by the matrix A, where the (I, j) position of A is Pi, j. We can easily calculate the t-order probability transfer matrix as follows:


(2) $$P_{I}\,\left(k|i\right)=\left|A^{I,K}\right|$$

where A is a probability matrix, and the sum of all rows is 1. The posterior probability distribution of node K on labels is easy to calculate as follows:


(3) $$P_{p}\,\left(y|i\right)=P\,\left(y|1\right)\,P_{p}\,\left(1|k\right)+P\,\left(y|2\right)\,P_{p}\,\left(2|k\right)+\ldots +P\,\left(y|i\right)\,P_{p}\,\left(i|k\right)$$

Then we can use the maximum posterior probability method to estimate the labels of nodes without labels:


(4) $$c_{k}=\arg\min p_{c}\,P\,\left(i|k\right)$$

### Research on the association between community psychological label and user portrait model

The association algorithm between community psychological labels and user portrait model is also based on a mainstream hypothesis in semi-supervised learning field, namely, the manifold hypothesis, which holds that labels of different nodes with similar distances are also similar under a certain metric criterion. Like the previous algorithm, we still need to define a weight matrix W between any two nodes (I, j), where the value of the matrix W for position (I, j) is defined as follows:


(5) $$w_{i\,k}=\exp\left(\sum_{i}{\left(y_{i}^{d}-y_{i}^{d}\right)}^{2}\right)/\delta^{2}$$

The association algorithm of community psychological label and user portrait model is used to describe the propagation process of the label in the network from the labeled node to the unlabeled node w. Similarly, we can define a probability transition matrix T in terms of the weight matrix L as follows:


(6) $$T_{L\,k}=w_{\mathrm{ik}}\,/\,\sum_{k}w_{i\,k}$$

The original network structure is transformed into a data structure suitable for the topic model. Therefore, before introducing the flowchart of the whole algorithm framework, how to transform the data structure of the social network into a data structure suitable for the topic model is shown in Figure 2.

**FIGURE 2:** Block diagram of association between community psychological label and user portrait model.

The first-order social relationship of each node in the social network corresponds to a document in the document set. Here, the first-order friend relationship is a super parameter and can be adjusted according to needs. All users in this first-order social relationship correspond to one word in the document; in addition, the label information known to each user is treated as the label information of the word in the document. Finally, the document’s own label can be set according to the label information of all words in the document. Generally, we default to the collection of all labels.

To further explore the relevance and explainability between themes and users’ Big Five personality traits, this study tries new methods. Considering that topics can be represented by the probability distribution of a series of words, users of social networks can also be represented by words in their own microblogs, and each topic can be regarded as a user of a social network. The next step is to find out the characteristics of the training model, predict each theme of the Big Five personality, and then look at the scores of subjects in each dimension of the Big Five personality so as to further find the correlation between theme and personality and interpretability. In this experiment, Linguistic Inquiry and Word Count (LIWC) of Sina Weibo users was used as the feature. In the experiment process, Chinese word segmentation is first carried out. During the process of word segmentation, LIWC dictionary should be added to ensure that the words in LIWC dictionary can be correctly cut. Then, LIWC features were extracted to obtain the LIWC features of 1,034 Sina Weibo users. Since the distribution of the theme word is in the form of probability, the algorithm of this experiment is different from the general word counting method of LIWC. In this experiment, the features of LIWC are normalized in the form of the proportion of the number of LIWC so as to match the features of the theme of LIWC.

Next, the five personality models are trained, respectively. The linear regression model of the five personality dimensions is used to predict the model. The model correlation coefficients are shown in Table 2, it can be seen that data sets in this experiment, compared with the theme as the characteristic of the Big Five personality model, besides the openness to experience O dimensions, the correlation coefficient of the rest of the dimensions are slightly higher. This also indicates that there is indeed a correlation between user’s writing language pattern and user’s personality.

**TABLE 2:** Correlation coefficients of the Big Five personality prediction model with linguistic inquiry and word count (LIWC) features.

	A	B	C	E	N
Correlation coefficient	0.0712	0.1334	0.1229	0.2123	0.1371

After obtaining a five-dimensional model, the experiment will focus on the subject’s “personality.” The topic at k = 60 extracted from the LDA topic model in the previous section is selected as the research object. The experiment needs to extract LIWC features from the topic vocabulary matrix of these 60 topics. Here, the extraction method of LIWC is different from the general one because the words under the topic are expressed in the form of probability and will not repeat. Therefore, the probability sum of words satisfying the LIWC category is taken as the LIWC feature of the subject of this experiment.

After extracting the LIWC features of the theme, the feature distribution was input into the five Big Five personality prediction models trained above to obtain the predicted personality scores of each theme. Table 3 is the statistical information corresponding to the Big Five A, B, C, E, N personality prediction score obtained from the topic of 50 dimensions.

**TABLE 3:** Statistical information of the 60-dimension subject Big Five personality prediction scores.

	A	B	C	E	N
Minimum value	17.98	9.96	3.23	15.26	3.56
Maximum	48.98	62.34	54.37	52.67	42.23
Average	31.58	27.82	24.45	34.67	25.89
Standard deviation	6.78	7.78	12.35	7.98	6.78

Of the Big Five, conscientiousness refers to the way we control, manage, and regulate our impulses. People with high conscientiousness tend to avoid trouble and achieve greater success. People who are highly conscientious are thought to be more intelligent and reliable, but highly conscientious people can be perfectionists or workaholics. Extremely conscientious individuals are perceived as dull, boring, and lifeless. Individuals with low conscientiousness are often perceived as happy, interesting, and good playmates. However, impulsive behavior often brings trouble to oneself. Although it brings temporary satisfaction to individuals, it is easy to produce long-term adverse consequences, such as attacking others and taking drugs.

When performing retrieval tasks, users upload retrieval data (text or image) and upload the uploaded data to the server through the query interface. After feature data processing, more hash codes and similarity calculation mode data in the database will be obtained and returned. The higher the similarity retrieval of results is, the original multimodal data after feature processing is stored in multimodal database. The calculation method of feature matching is to compare the input hash code of the data to be retrieved with the hash code in the database to calculate the similarity one by one, and then return the required result. After feature extraction and hash code generation, all feature vectors obtained are transformed into hash codes, so there are many commonly used similarity calculation methods for hash codes, such as Euclidean distance and Mahalanobis distance.

## Example verification

For the MIRFLICKR-50K data set, we randomly selected 10,000 instances as the training set. For testing, we used 2,000 instances of this data set as the test set and the rest as the retrieval set. For the NUS-wide data set, 10,500 data points were randomly sampled as the training set. For testing, we used 2,100 instances of this data set as the test set and the rest as the retrieval set. The Alexnet network has been pre-trained on the ImageNet data set and fine-tuned as we train our model. In the experiment, we will take/ = 0.3 and u = 0.1. In addition, the batch size is fixed at 128, and the algorithm can be run 500 times.

The performance of all comparison methods in our experiment was directly evaluated using average accuracy and accuracy recall curves, as shown in Table 4 and Figures 3, 4.

**TABLE 4:** Average accuracy (RP) of each method.

Task	Method	MIRFL-50K			NUS-wide		
		16 bits	32 bits	64 bits	16 bits	32 bits	64 bits
Image to text	KQDH	0.723	0.783	0.745	0.634	0.634	0.678
	DCMH	0.734	0.734	0.723	0.632	0.612	0.657
	SCM	0.635	0.653	0.643	0.487	0.489	0.498
	STMH	0.583	0.589	0.589	0.438	0.453	0.345
	LSSH	0.578	0.578	0.581	0.398	0.389	0.423
	CVH	0.612	0.612	0.613	0.387	0.378	0.378

**FIGURE 3:** Accuracy recall rate curve of MIRFLICKR-50K data set.

**FIGURE 4:** Accuracy recall rate curve of NUS-WEE data set.

Users on Facebook’s data set have many different attributes, including where they live, education, gender, hometown, and language. These user attributes were recommended when we first registered to use Facebook. However, most of the time we did not fill in the complete information, but only filled in part of the information selectively, which is also in line with human nature. As for the data set we used, we made a detailed statistics of user attribute information related to this data set. Table 5 presents the completeness of users’ filling in different attributes in the Facebook data set we used. It can be seen intuitively that many user attributes are incomplete. Only 15.0% of the attributes with the lowest filling proportion (such as gender and place of work) are complete, while only 66.7% of the attributes with the highest filling proportion (such as educational background) are complete. Many of the attributes we care about that are closely related to practical applications (such as place of residence and age) were completed with 41.1% or less.

**TABLE 5:** Completeness of each attribute information in the Facebook data set.

Attribute	Number of labeled users	Fraction
Gender	607	15.2%
Location	1,657	42.1%
Education	2,694	66.8%
Language	742	18.7%
Age	572	39.2%
Work-location	603	14.5%
Hometown	1,056	26.5%

Figure 5 describes the degree (number of friends) distribution of each node (user) in the network. We can see that this distribution is actually a heavy-tailed power law distribution, and the degree of most nodes is in the range [0, 200]. This distribution is also in line with our common sense of social networks. Generally speaking, most users in a social network are ordinary users with less than 100 friends, and only a few users have a large number of friends or fans. The degree of users is in the interval [0, 50], and the problem of attribute loss of this group of users is more serious than that of users in other intervals.

**FIGURE 5:** Statistical analysis of residence attributes in the Facebook data set.

Combined with the advantages of neural network model, the effect of user population attribute prediction task has been further improved. The improved DOC2VEC-QDV model has the best effect. This is because in the improved DDBOW-QDV training mode, the bigRAM characteristics of query words such as word segmentation and splicing are carried out on users’ query words, which can make up for the neglect of context information in the original training mode, thus improving the overall effect of the model. However, in dM-QDV training mode, only focus on the internal connection of query words, which can reduce the complexity of the model. The two training modes complement each other and finally improve the performance of the model. The bar chart of comparison of various models is shown in Figure 6.

**FIGURE 6:** Bar chart of comparison of various models.

The neural network model based on the multi-modal user portrait algorithm has better classification accuracy for age and degree labels than for gender labels. This is because many modal model, neural network algorithm in the first hierarchy model for classification task, more able to output the probability of each category. Based on the first-level model, the threshold judgment and mutual verification of the second-level model can make better use of the correlation between user group attributes to learn the second-level model, so that the feature fusion effect of multiclassification tasks is better. Finally, the user portrait algorithm based on Stacking strategy and XGBoost is verified, which can better fuse features and improve classification accuracy. Compared with the BDCC algorithm, Ensemble algorithm is found to be slightly worse than the model proposed in this article, which again shows that the prediction effect of user portrait algorithm based on Stacking strategy and XGBoost on user population multidimensional attribute tags is improved, proving the effectiveness of the proposed algorithm model. The histogram of model comparison is shown in Figure 7.

**FIGURE 7:** Bar chart of comparison between different models.

The experiment verified the validity of the model through the classification prediction of gender, age, and education background labels on the test set, and counted the accuracy and average accuracy of the three labels, as shown in Table 6.

**TABLE 6:** Classification prediction results of different models.

Model	Education	Age	Sex	Ave
BERT	68.83	62.82	84.05	71.92
BDCC	67.83	64.13	86.22	72.75
Ensemble	71.05	65.72	86.45	74.46
BERT-ensemble	71.22	66.15	86.52	74.62

## Conclusion

To obtain better results in multidimensional population attribute label prediction tasks, a user profiling algorithm based on Stacking strategy and XGBoost is proposed. At the first level of the whole algorithm, the user attribute features are obtained from different angles by combining different types of basic models, and then the association information between user attribute features is obtained by using multimodal neural network strategy to complete the prediction of user group attribute tags. Experiments show the effectiveness of the algorithm. Secondly, word-level supervision information is introduced to control the probability of each topic being assigned to the word, which ultimately improves the prediction accuracy of the model. To further improve the prediction performance of the model, the final structure of the algorithm model based on the association between the community psychological label and the user portrait model is used to refine the model. Finally, experiments on real social network data sets verify the accuracy of the proposed algorithm in predicting user attributes and the potential relevance formed by friend relationships between users, and verify the robustness of the model by predicting different types of attributes. The next step is to divide the dimensions from the perspective of context. The attributes of the conceptual model of user portrait are mined from the five dimensions of user context, project context, time context, space context, and computing context, and the concept lattice method is introduced to realize the construction of user portrait.

## Data availability statement

The original contributions presented in the study are included in the article/supplementary material, further inquiries can be directed to the corresponding author.

## Ethics statement

Ethical review and approval was not required for the study on human participants in accordance with the local legislation and institutional requirements. Written informed consent from the patients/participants OR patients/participants legal guardian/next of kin was not required to participate in this study in accordance with the national legislation and the institutional requirements.

## Author contributions

Both authors listed have made a substantial, direct, and intellectual contribution to the work, and approved it for publication.

## References

[B1] AkbarH.ZahraH.AwatF. (2017). Association of stressful life events with psychological problems: A large-scale community-based study using grouped outcomes latent factor regression with latent predictors. *Comput. Math. Methods Med.* 2017 21–32. 10.1155/2017/3457103 29312459PMC5625761

[B2] Carhart-HarrisR. L.BolstridgeM.RuckerJ. (2016). Psilocybin with psychological support for treatment-resistant depression: An open-label feasibility study. *Lancet Psychiatry* 3 542–557. 10.1016/S2215-0366(16)30065-727210031

[B3] HoJ.NgaiS. P. C.WuW. K. (2018). Association between daily life experience and psychological well-being in people living with nonpsychotic mental disorders. *Medicine* 97:e9733. 10.1097/MD.0000000000009733 29369215PMC5794399

[B4] JaimeD.KimD. J.MikeL. (2018). Feedback-informed treatment versus usual psychological treatment for depression and anxiety: A multisite, open-label, cluster randomised controlled trial. *Lancet Psychiatry* 5 564–572. 10.1016/S2215-0366(18)30162-7 29937396

[B5] JimenezG. C.EissaS.NgA. (2015). Aptamer-based label-free impedimetric biosensor for detection of progesterone. *Anal. Chem.* 87 872–889. 10.1021/ac503639s 25486123

[B6] KayserS.BewernickB. H.MatuschA. (2015). Magnetic seizure therapy in treatment-resistant depression: Clinical, neuropsychological and metabolic effects. *Psychol. Med.* 45 1073–1092. 10.1017/S0033291714002244 25420474

[B7] KhalafA.NabianM.FanM. (2020). Analysis of multimodal physiological signals within and between individuals to predict psychological challenge vs. threat. *Expert Syst. Appl.* 140:112890. 10.1016/j.eswa.2019.112890

[B8] LiM.KongD.ChaoY. Y. (2020). Association between personality traits and elder abuse in a community-dwelling Chinese population: Findings from the PINE study. *J. Elder Abuse Negl.* 32 317–333. 10.1080/08946566.2020.1782300 32580693

[B9] LindenT.JongJ. D.LuC. (2021). An explainable multimodal neural network architecture for predicting epilepsy comorbidities based on administrative claims data. *Front. Artif. Intell.* 4:610197. 10.3389/frai.2021.610197 34095818PMC8176093

[B10] LiuT.KongJ.JiangM. (2019). RGB-D action recognition based on discriminative common structure learning model. *J. Electron. Imaging* 28:023012. 10.1117/1.JEI.28.2.023012

[B11] LudwinK.CapstickA. (2015). Using participatory video to understand diversity among people with dementia in long-term care. *J. Psychol. Issues Organ. Cult.* 5 30–38. 10.1002/jpoc.21161

[B12] MiquelM. J.CaplliureE. M.PerezC. (2017). Buying private label in durables: Gender and other psychological variables. *J. Retail. Consum. Serv.* 34 349–357. 10.1016/j.jretconser.2016.07.013

[B13] MurayamaY.OhyaA. (2021). A cross-sectional examination of the simultaneous association of four emotion regulation strategies with abnormal eating behaviours among women in Japan. *J. Eat. Disord.* 9 3241–3256. 10.1186/s40337-021-00477-7 34583776PMC8480045

[B14] RathiN.RoyK. (2018). STDP based unsupervised multimodal learning with cross-modal processing in spiking neural network. *IEEE Trans. Emerg. Top. Comput. Intell.* 8 121–132.

[B15] ShelefA.BarakY.BergerU. (2016). Safety and efficacy of medical cannabis oil for behavioral and psychological symptoms of dementia: An-open label, add-on, pilot study. *J. Alzheimers Dis.* 51 15–19. 10.3233/JAD-150915 26757043

[B16] SolowijN.BroydS. J.BealeC. (2018). Therapeutic effects of prolonged cannabidiol treatment on psychological symptoms and cognitive function in regular cannabis users: A pragmatic open-label clinical trial. *Cannabis Cannabinoid Res.* 3 21–45. 10.1089/can.2017.0043 29607408PMC5870061

[B17] SteinerB. E.PeschelA. O.GrebitusC. (2017). Multi-product category choices labeled for ecological footprints: Exploring psychographics and evolved psychological biases for characterizing latent consumer classes. *Ecol. Econ.* 140 251–264. 10.1016/j.ecolecon.2017.05.009

[B18] SuX.WongV.LiangK. A. (2021). Multilevel investigation of the association between collective psychological ownership as psychosocial resources and social workers’ turnover intention. *Br. J. Soc. Work* 5 287–304. 10.1093/bjsw/bcab245

[B19] WeiWeiQ. (2020). Multi-modal facial expression feature based on deep-neural networks. *J. Multimodal User Interfaces* 14 17–23.

[B20] WilliamsJ.BucciS.BerryK. (2018). Psychological mediators of the association between childhood adversities and psychosis: A systematic review. *Clin. Psychol. Rev.* 65 1650–1673. 10.1016/j.cpr.2018.05.009 30243100

[B21] ZhengY.ZhangY. J.LarochelleH. A. (2016). Deep and autoregressive approach for topic modeling of multimodal data. *IEEE Trans. Pattern Anal. Mach. Intell.* 38 1056–1069. 10.1109/TPAMI.2015.2476802 26372202

